The article "Translation and Initial Validation of the Chinese (Cantonese) Brief 2-Way Social Support Scale for Use in People with Chronic Stroke" was published in 2022. Journal: Biomed Res Int.

# Translation and Initial Validation of the Chinese (Cantonese) Brief 2-Way Social Support Scale for Use in People with Chronic Stroke

**DOI:** 10.1155/2022/3511631

**Published:** 2022-06-29

**Authors:** Tai Wa Liu, Shamay S. M. Ng, Joshua Tsoh, Peiming Chen, Richard H. Xu, Thomson W. L. Wong, Mimi M. Y. Tse

**Affiliations:** ^1^School of Nursing and Health Studies, Hong Kong Metropolitan University, Ho Man Tin, Hong Kong; ^2^Department of Rehabilitation Sciences, The Hong Kong Polytechnic University, Hung Hom, Hong Kong; ^3^Department of Psychiatry, Prince of Wales Hospital & Shatin Hospital, Sha Tin, Hong Kong; ^4^School of Nursing, The Hong Kong Polytechnic University, Hung Hom, Hong Kong

## Abstract

**Background:**

Social support is important for stroke rehabilitation. Conventionally, social support is evaluated from the level of support received. However, the bidirectional support hypothesis postulated that self-perceived social support is optimized if individuals provide and receive social support in a balanced manner. The Brief 2-Way Social Support Scale (Brief 2-Way SSS) is a social support instrument measuring the reciprocity of receiving and giving emotional and instrumental social support.

**Objective:**

(1) To translate and culturally adapt the English version of the Brief 2-Way SSS into Chinese (Cantonese) (Brief 2-Way SSS-C), (2) to report the results of validation of the Brief 2-Way SSS-C, and (3) to investigate the level of social support in people with stroke in Hong Kong.

**Methods:**

The Brief 2-Way SSS-C was produced following the standard forward-backward translation model. People with stroke (*n* = 109) and age-matched controls (*n* = 53) were recruited through a university-affiliated neurorehabilitation laboratory.

**Results:**

The Brief 2-Way SSS-C demonstrated excellent content validity, acceptable to good internal consistency (Cronbach's alpha of 0.74–0.88), and good test-retest reliability (intraclass correlation coefficient of 0.76–0.81). There were no ceiling or floor effects, and the MDC95 across all subscales was 4. The Brief 2-Way SSS-C subscales had significant correlations with various health-related outcome measures. People with stroke had a lower level of social support than the age-matched healthy controls.

**Conclusions:**

The Brief 2-Way SSS-C is a culturally relevant, reliable, and valid outcome measure for the level of social support in community-dwelling people with stroke.

## 1. Introduction

Social support can be defined as any support given outside formal settings, such as by relatives or friends instead of health professionals or social services providers, and can be applied in both directions; i.e., a person can both receive and provide social support [1, 2]. Conventionally, social support is evaluated from the emotional and instrumental aspects [3]. Emotional support involves the provision of care, love, acceptance, and encouragement. It has been shown to reinforce self-esteem, induce feelings of being cared about and valued, and enhance emotional well-being. Instrumental support is generally more quantifiable and includes elements, such as assistance with daily chores, that help the receiver feel more able to meet the demands of daily living and enhance their self-esteem in the long run [4–7]. Social support can protect against a significant decline in functional mobility in the elderly [8]. A systematic review of 78 studies with a combined sample size of 118,932 older adults, focusing on factors causing functional status decline, found that a low level of social support was associated with limitations in functional mobility [9]. Another study found that older adults with a high level of emotional support had a lower occurrence of physical disability (odds ratio [OR] = 0.62, *p* < 0.001) [8] and lower dependency on activities of daily living (ADL) (adjusted OR = 0.21) [10].

However, the role of social support in stroke rehabilitation may have been underestimated. In people with stroke, a higher level of social support correlates with a better functional capacity [11–13], lower levels of depression [13], and improved social participation [13], mood [13], and ADL [11–13]. Glass and Maddox and Glass et al. [11, 12] found that social support, as measured by the Inventory of Socially Supportive Behaviors, was significantly (*p* < 0.05) related to the recovery of functional capacity and ADL, as measured by the Barthel Index (BI), in 46 and 44 people with stroke, respectively. Tsouna-Hadjis et al. [13] found that in a sample of 43 people with stroke, those with a high level of social support from family members, as measured by the Family Social Support Scale, had significantly (*p* < 0.05) better functional capacity and ADL as measured by the BI, lower levels of depression as measured by the Zung Scale, a higher level of social participation as measured by the General Health Questionnaire Index (GHQI) Subscale A, and lower levels of anxiety and insomnia as measured by the GHQI Subscales B and C. Social support can enhance self-esteem and motivation for rehabilitation in people with stroke. The receipt of social support and the observation of their own recovery also reinforce stroke survivors' efforts to recover [14].

A low level of social support has been reported in people with stroke [15]. Lima et al. [15] revealed that 74.1% of 108 people with sequelae of chronic stroke presented with low-to-medium received social support, as measured by the Medical Outcomes Study Social Support Survey. As the level of social support affects the functional mobility and rehabilitation outcome of people with stroke, a reliable and valid outcome measure for documenting the level of social support in Chinese people with stroke is needed.

The 2-Way Social Support Scale (2-Way SSS) is a validated, 4-factor, 20-item instrument that measures the reciprocity of emotional and instrumental social support [1] . Each item is measured on a 6-point Likert scale ranging from 0 (not at all) to 5 (always) [1] . A higher score represents a higher level of giving or receiving social support. The 20-item scale has good internal consistency and predictive validity and fair convergent validity. To enhance the feasibility of clinical use, the Brief 2-Way SSS, with 4 factors but just 12 items, was developed and tested in a group of elderly individuals [16].

Although the Brief 2-Way SSS is a useful outcome measure for assessing social support in the general population, it has not been validated in people with stroke. The scale has also not been translated from English to Chinese (Cantonese), which is more culturally accessible to the Hong Kong Chinese population, nor has it been tested in Chinese (or any Asian) settings. No study has investigated the psychometric properties of the Brief 2-Way SSS in people with stroke, and the level of social support in people with stroke in Hong Kong is understudied. Therefore, the objectives of this study were (1) to translate and culturally adapt the English version of the Brief 2-Way SSS into Chinese (Cantonese) (Brief 2-Way SSS-C); (2) to report the results of initial validation of the Brief 2-Way SSS-C including the internal consistency, test-retest reliability, minimal detectable change (MDC), and correlations in community-dwelling people with stroke in a Chinese community setting; and (3) to investigate the level of social support in community-dwelling people with stroke in Hong Kong.

## 2. Methods

### 2.1. Translation

The translation and cross-cultural adaptation of the Brief 2-Way SSS were based on the standard forward-backward translation model [17]. Two independent bilingual translators (one a professional translator with no background in medicine or rehabilitation, the other a physiotherapist with more than 6 years of clinical experience), both with Chinese (Cantonese) as their mother language, translated the original English version of the Brief 2-Way SSS into separate initial drafts in Chinese (Cantonese) (D1 and D2). D1 and D2 and the original English version of the Brief 2-Way SSS were reviewed by the same two translators, and all discrepancies identified between D1 and D2 were resolved by discussion to reach a consensus version (D1-2). Then, another two independent translators who were blinded to the original Brief 2-Way SSS back-translated D1-2 into English independently. As no conceptual discrepancies were identified between the backward translations, D1-2 was adopted as the Chinese (Cantonese) version of the Brief 2-Way SSS and evaluated by an expert panel of three experienced registered physiotherapists, one experienced rehabilitation therapist, one experienced registered nurse, and one experienced registered mental health nurse for equivalence of content, semantics, conceptual properties, and any technical discrepancies with the original English version. The version they produced was named the Chinese (Cantonese) 2-Way SSS-Pilot and was piloted in a convenience sample of 10 community-dwelling people with stroke to ascertain clarity and comprehensibility. As no amendment was required, the final version, denoted the Brief 2-Way SSS-C, was confirmed.

### 2.2. Sample and Data Collection Procedure

A total of 109 people with stroke and 53 age-matched healthy older people were recruited through a university-affiliated neurorehabilitation laboratory using poster advertisements (Table 1). The inclusion criteria for stroke subjects were as follows: being 50 years old or above, having suffered a single stroke at least 1 year before the start of the study, having an abbreviated mental test score of 7 or above, being able to understand Cantonese, and being able to independently walk 10 m with or without walking aids. The exclusion criteria comprised having any other comorbid neurological diseases (e.g., Parkinson's disease) or having unstable medical conditions, such as cardiovascular problems, that might affect the validity of the assessment. For healthy subjects, the inclusion and exclusion criteria were the same except that a history of stroke was not among the inclusion criteria.

All of the assessments were conducted in a university-affiliated neurorehabilitation laboratory. The subjects were informed about the objectives and procedures of the study and asked to give their consent before participating in the tests. Sociodemographic data were then collected from all 109 stroke subjects using a questionnaire. The Brief 2-Way SSS-C, the Fugl-Meyer Assessment of Lower Extremity (FMA-LE), the Timed Up-and-Go Test (TUGT), the Chinese version of the Community Integration Measures (CIM-C), and the Chinese version of the 12-item Short Form Survey (SF-12-C) were administered to all subjects. The order of the tests was determined randomly by drawing lots, and at least 2 minutes of rest was allowed between the tests to minimize fatigue. One week later, 63 of the 109 stroke subjects, who were randomly selected by drawing lots, were reassessed with the Brief 2-Way SSS-C to establish test-retest reliability. The healthy subjects were assessed with the Brief 2-Way SSS-C only once.

For the sample size calculations, an alpha level of 0.05 (2-tailed) and a power of 0.80 were adopted. To avoid an overestimation of the consistency of Brief 2-Way SSS-C in the stroke subjects, the expected test-retest reliability was set at an intraclass correlation coefficient (ICC) = 0.50. The required sample size was therefore calculated as 22 [18]. Allowing for 20% attrition, the total minimum sample size was calculated as 27 ( = 22 + 20%of 22).

The protocol was approved by the Departmental Research Committee of The Hong Kong Polytechnic University and conducted according to the principles of the Declaration of Helsinki for human experiments.

### 2.3. Outcome Measures

#### 2.3.1. The Chinese Version of the Brief 2-Way Social Support Scale (Brief 2-Way SSS-C)

The Brief 2-Way SSS-C contains 12 items to measure the respondent's receipt and giving of emotional and instrumental support. All items are rated on a 6-point Likert scale from 0 (not at all) to 5 (always). The total score ranges from 0 to 72, with a higher score indicating a higher level of giving or receiving social support. The original Brief-2-Way SSS has demonstrated good internal consistency (Cronbach's alpha = 0.75–0.88) [1, 16] and moderate test-retest reliability (ICC = 0.69–0.73) [16] in healthy subjects. The Brief 2-Way SSS showed a better fit to the data than the original scale (20-item: comparative fit index (CFI) = 0.90, 12-item: CFI = 0.97) [16] and also has excellent internal consistency (Cronbach's alpha = 0.75–0.88) and satisfactory test-retest reliability (3-month interval; *r* = 0.69–0.73) [16].

#### 2.3.2. Fugl-Meyer Assessment of Lower Extremity (FMA-LE)

The FMA-LE is a 17-item scale developed to assess the movement, coordination, and reflex action of the hip, knee, and ankle [19]. Subjects' ability to complete each item is assessed on a 3-point ordinal scale, with 0 points representing inability to perform, 1 point representing ability to perform partially, and 2 points representing ability to perform fully compared with the nonlesion side, with a maximum possible score of 34. A higher FMA-LE score indicates a better motor function of the lower extremity. It has excellent internal consistency (Cronbach's alpha = 0.94) and good test-retest reliability (ICC = 0.87) in people with stroke [20, 21].

#### 2.3.3. The Timed Up-and-Go Test (TUGT)

The TUGT is a measure of functional ability, which evaluates the subject's fall risk, balance ability, sit-to-stand ability, and walking ability. The TUGT's simple and time-efficient nature makes it a widely used measure in clinical and research settings. The psychometric properties of the TUGT have been validated in community-dwelling older adults. It has excellent interrater reliability (ICC_3,3_ = 0.98) and moderate test-retest reliability (ICC = 0.56) [22].

#### 2.3.4. The Chinese Version of the Community Integration Measure (CIM-C)

The CIM-C is a 10-item scale developed to measure subjects' community participation after brain injury in terms of “relationship and engagement,” “sense of knowing,” and “independent living” and has been validated in Chinese people with stroke. All items are rated on a 5-point Likert scale from 1 (always disagree) to 5 (always agree). The total score ranges from 10 to 50, with a higher score indicating better community integration. The CIM-C has demonstrated good internal consistency (Cronbach's alpha = 0.84) and test-retest reliability (ICC = 0.84, 95% confidence interval (CI) = 0.64–0.93) in people with chronic stroke [23].

#### 2.3.5. The Chinese Version of 12-Item Short Form Survey (SF-12-C)

The SF-12-C measures subjects' physical (physical component summary, PCS) and mental (mental component summary, MCS) health-related quality of life. The instrument evaluates eight subscales relating to health-related quality of life: physical functioning, role (physical), bodily pain, general health, vitality, social functioning, role (emotional), and mental health [24]. It has demonstrated good internal consistency (Cronbach's alpha of PCS = 0.67; MCS = 0.60) and good test-retest reliability (ICC of PCS = 0.82; MCS = 0.81) in healthy Chinese adults [25].

### 2.4. Statistical Analysis

Quantitative data were analyzed using Statistical Package for the Social Sciences (SPSS) (version 26). The significance level was set at 0.05. The normality of the sample data was evaluated by the Shapiro-Wilk test. The internal consistency was measured by Cronbach's alpha. The test-retest reliability was measured by ICC_3,1_ with an optimal between measurement correlation score of 0.70. ICCs of >0.9, 0.75–0.90, 0.50–0.75, and<0.50 indicate excellent, good, moderate, and poor correlation, respectively [26]. The MDC was calculated based on the test-retest reliability (ICC_3,1_) and the standard error of measurement (SEM) using the following formula: MDC_95_ = 1.96 × SEM × √(2), where SEM = SD × √(1 − ICC_3,1_) and SD is the standard deviation. The presence of a floor or ceiling effect was defined as >15% of subjects achieving the lowest or highest score, respectively. Correlations between the Brief 2-Way SSS-C score and the FMA-LE, TUGT, CIM-C, and SF-12-C scores were examined using Pearson's *r* and Spearman's rho for normally and nonnormally distributed variables, respectively. Correlation strength was defined as weak (<0.25), fair (0.25–0.50), moderate to good (0.50–0.75), and good to excellent (>0.75) [27].

## 3. Results

### 3.1. Content Validity

All items on the Brief 2-Way SSS-C demonstrated an acceptable item-level content validity index (CVI) (I-CVI) (I − CVI ≥ 0.0.78) [28] except for item 5 (Table 2). The mean scale-level CVI (S-CVI/Ave) was 0.97, and the proportion of universal agreement (UA) of the expert panel members (S-CVI/UA) was 0.92, suggesting that the Brief 2-Way SSS-C has excellent overall scale-level content validity [29].

### 3.2. Characteristics of the Subjects

There were 63 male and 46 female stroke subjects with a mean age of 63.63 years (SD = 6.24 years) (Table 1). Their mean duration since stroke was 6.58 years (SD = 4.30 years); 49 (45%) of them had left-side hemiplegia and 60 (55%) had right-side hemiplegia. Twenty-four (22%) were educated to primary school level or below, 70 (64%) had completed secondary school and 15 (14%) were educated to college level or above. The majority (*n* = 75, 69%) had a history of ischemic stroke, and 34 (31%) had a history of hemorrhagic stroke. Ten stroke subjects (9%) were living alone, and 99 (91%) were living with family members or carers. Concerning marital status, 11 (10%) were single, 81 (74%) were married, 9 (8%) were divorced or separated, and 8 (7%) were widowed.

### 3.3. Internal Consistency

The Brief 2-Way SSS-C subscales demonstrated acceptable to good internal consistency (0.74–0.88) (Table 3). The item-total correlations were moderate to good, ranging from 0.52 (item 8) to 0.82 (item 9) in the subscales. No item-deletion could improve the Cronbach's alpha values in any of the subscales.

### 3.4. Test-Retest Reliability, MDC, and Ceiling and Floor Effects

Sixty-seven of the stroke subjects participated in the reassessment after a 1-week interval. The Brief 2-Way SSS-C demonstrated moderate to good subscale test-retest reliability, as reflected in the ICC_3,1_ values of 0.76 (95% CI = 0.64–0.84), 0.77 (95% CI = 0.65–0.85), 0.81 (95% CI = 0.70–0.88), and 0.78 (95% CI = 0.67–0.86) for the receiving emotional support, giving emotional support, receiving instrumental support, and giving instrumental support subscales, respectively (Table 4). The ICC values for the individual items ranged from 0.59 to 0.79, with item 3 (“People confide in me when they have problems”) showing the highest consistency (ICC_3,1_ = 0.79, 95% CI = 0.68–0.87). Item 11 (“I have someone to help me if I am physically unwell”) showed the lowest consistency (ICC_3,1_ = 0.59, 95% CI = 0.40–0.72). The MDC_95_ (SEM) of the subscales of receiving emotional support, giving emotional support, receiving instrumental support, and giving instrumental support was 3.23 (1.17), 3.75 (1.36), 3.59 (1.30), and 3.43 (1.24), respectively. No item had more than 15% of subjects scoring the lowest or highest item score.

### 3.5. Correlations between the Brief 2-Way SSS-C and Variables of Interest

The receiving subscales had significant weak to fair correlations with the FMA-LE (receiving emotional support, *r* = 0.21, *p* = 0.028; receiving instrumental support, *r* = 0.23, *p* = 0.016), CIM-C (receiving emotional support, *r* = 0.31, *p* = 0.001; receiving instrumental support, *r* = 0.39, *p* < 0.001), and MCS-C (receiving emotional support, *r* = 0.25, *p* = 0.008; receiving instrumental support, *r* = 0.28, *p* < 0.001) scores (Table 5). The giving subscales had significant weak to fair correlations with the FMA-LE score (giving emotional support, *r* = 0.36, *p* < 0.001; giving instrumental support, *r* = 0.36, *p* < 0.001), TUGT completion time (giving emotional support, *r* = −0.22, *p* = 0.024; giving instrumental support, *r* = −0.39, *p* < 0.001), CIM-C (giving emotional support, *r* = 0.45, *p* < 0.001; giving instrumental support, *r* = 0.46, *p* < 0.001), PCS-C (giving emotional support, rho = 0.22, *p* = 0.023; giving instrumental support, rho = 0.36, *p* < 0.001), and MCS-C (giving emotional support, *r* = 0.22, *p* = 0.023; giving instrumental support, *r* = 0.35, *p* < 0.001). The Brief 2-Way SSS-C items had no ceiling or floor effects.

Table 6 compares the main Brief 2-Way SSS-C subscale scores between the stroke subjects and healthy subjects. The healthy subjects scored higher on the subscales of receiving emotional support (*t* = −3.61, *p* = 0.001), giving emotional support (*t* = −3.85, *p* < 0.001), receiving instrumental support (*t* = −2.14, *p* = 0.04) and giving instrumental support (*t* = −5.77, *p* < 0.001).  Table 7 summarizes the mean score for each Brief 2-Way SSS-C subscale according to various selected demographics of the stroke subjects. The independent *t*-test and one-way ANOVA revealed no significant differences in any of the Brief 2-Way SSS subscale scores of the stroke subjects when stratified by sex, education level, marital status, or living arrangement. However, there were significant differences in the giving emotional support (*t* = −3.27, *p* = 0.003) and giving instrumental support (*t* = −3.08, *p* = 004) subscale scores between stroke subjects with high mobility function (FMA-LE score ≥ 21) and low mobility function (FMA-LE score < 21) [30].

## 4. Discussion

This is the first study to investigate the psychometric properties of the Brief 2-Way SSS-C among people with stroke. The Brief 2-Way SSS-C subscales showed acceptable to good internal consistency, good test-retest reliability, and weak to fair associations with a lower limb impairment measure (FMA-LE), a functional ability measure (TUGT), a community reintegration measure (CIM-C), and a health-related quality of life measure (SF-12-C). Moreover, we attempted to expand the understanding of self-perceived social support of people with stroke using an instrument developed on the basis of the bidirectional support hypothesis [31], in which psychological benefits are believed to be optimized if individuals provide and receive support in a balanced manner [32, 33].

In this study, we established the cultural equivalence of the Brief 2-Way SSS, as reflected by the good item-level content validity except for item 5 (“I give others a sense of comfort in times of need”) and excellent scale-level content validity. During the translation process, our professional translators disagreed on the wording of item 5 as the English term “a sense of comfort” can be expressed in various formal and informal ways in Cantonese. With the consensus reached by our expert panel, this semantic difference between the original English version and the Chinese (Cantonese) version was resolved before producing the pilot Chinese (Cantonese) version.

We calculated the Cronbach's alpha coefficients for all of the Brief 2-Way SSS-C subscales to evaluate the internal consistency at the subscale level and item level, i.e., the ability to measure the same traits of the concerned construct. The acceptable to good Cronbach's alpha values of the Brief 2-Way SSS-C subscales (0.74 to 0.88) were comparable to those of the original Brief 2-Way SSS (ranging from 0.75 to 0.90). The individual Brief 2-Way SSS-C items demonstrated good item-total correlations (*r* > 0.50). The Cronbach's alpha values of all of the Brief 2-Way SSS-C subscales were above 0.70 and below 0.90 [34], which suggested that no individual item of the Brief 2-Way SSS-C is redundant and all of the items measure the construct of self-perceived social support.

The good test-retest reliability of the Brief 2-Way SSS-C subscales (ICC = 0.76–0.81) is superior to those reported in the original study of the full version (*r* = 0.69–0.73) [16], indicating a high degree of repeatability for clinical use. One possible explanation for the good test-retest reliability is that we used a single examiner and adopted a shorter test-retest interval (1 week) than that adopted in the original study (3 months). It is believed that a 1-week interval for test-retest reliability can minimize the possibility of significant events in the interim while excluding memory effects. Moreover, the SEM values of the receiving emotional support, giving emotional support, receiving instrumental support, and giving instrumental support subscales were 7.8%, 9.1%, 8.7%, and 9.4%, respectively. These findings established the reliability of the Brief 2-Way SSS-C for use in ambulatory and cognitively intact community-dwelling chronic stroke survivors.

No previous study had established the MDC for the Brief 2-Way SSS-C. In this study, we established that a change of 4 points on each Brief 2-Way SSS-C subscale is needed to be 95% confident that true change has occurred. Establishing the MDC provides clinicians with a reference value to determine whether the extent of change in social support will have meaningful effects on people with stroke. Moreover, no ceiling or floor effects of the Brief 2-Way SSS-C were noted in this study. This indicates that the Brief 2-Way SSS-C can detect the variance in receiving and giving social support among community-dwelling people with chronic stroke without attenuation on either end of the scale.

As expected, the levels of functional ability, community integration, and mental health-related quality of life were significantly correlated with both the giving and receiving of social support. This is consistent with the previous findings that social support is associated with psychological and physical health among older people [8]. Taking into account the adverse consequences of stroke, we also examined the lower limb impairment and physical health-related quality of life of people with stroke. Our analysis identified that (i) the stroke-related functional impairment only related to the giving subscale but not the receiving subscale of the Brief 2-Way SSS-C and (ii) there were weak associations between social support with lower limb impairment and functional impairment and moderate association between social support with health-related quality of life, respectively. There are two possible explanations of this observed phenomenon. First, we believe that stroke-related functional impairment can adversely affect the self-rated readiness and ability to offer help to others but not to receive support from others. Thus, there was no significant correlation identified between the stroke-related functional impairment and level of receiving social support in this cohort of people with stroke. Secondly, although it is believed that people with physical disability and cognitive impairment could attract more social support, our study participants were recruited from the community through advertisements. They were socially active and probably had developed the compensatory and adaptive community living skills years after stroke. For this cohort of cognitively intact and socially engaged community-dwelling people with chronic stroke, their lower limb impairment and functional impairment may have less prominent roles in the perceived level of social support. Nonetheless, the perceived level of social support continued to exert significant influences on the health-related quality of life of people with chronic stroke.

Our findings were consistent with those of Lima et al. [15] that people with stroke had lower levels of social support than age-matched and marital status-matched healthy people. Moreover, our findings revealed that study participants with better levels of lower limb function had higher levels of self-perceived giving of social support than those with poorer lower limb function. It is reasonable to hypothesize that community-dwelling stroke survivors with minimal to mild levels of lower limb impairment were more able to integrate into the community and more willing to offer both emotional and instrumental social support than those with moderate to serious levels of lower limb impairment.

It is important to note that the psychometric properties of the Brief 2-Way SSS-C were established using a sample of ambulatory and cognitively intact community-dwelling chronic stroke survivors. Therefore, the findings may not be generalizable to those with more severe stroke-related impairments or in different phases of stroke and are limited to those fulfilling our inclusion and exclusion criteria. Moreover, women tend to be more able to maintain social networks than men. Due to the uneven male-female ratio in this study (63 : 46), we may have underestimated the level of social support in people with stroke.

## 5. Conclusion

Enhancing social support is a feasible way to improve the rehabilitative outcomes of people with stroke. Adaptation of a validated instrument can help quantify social support across cultures. In addition to producing a reliable and valid social support measure, our findings suggest that people with stroke have lower levels of giving support than receiving support. To optimize the level of social support, recovery, community reintegration, and quality of life, policymakers and clinicians could consider strategies to maximize the support-giving role of community-dwelling chronic stroke survivors.

## Figures and Tables

**Table 1:** Characteristics of participants.

	Stroke participants (*n* = 109)	Healthy participants (*n* = 53)
Age (y), mean (SD)	63.63 (6.24)	61.74 (7.39)
Sex, *n* (%)		
Women	46 (42.2)	38 (71.7)
Men	63 (57.8)	15 (28.3)
BMI (kg/m^2^), mean (SD)	23.96 (3.02)	22.59 (3.09)
Education level, *n* (%)		
Primary or below	24 (22.0)	9 (17.0)
Secondary	70 (64.2)	36 (67.9)
College or above	15 (13.8)	8 (15.1)
Marital status, *n* (%)		
Single	11 (10.1)	7 (13.2)
Married	81 (74.3)	45 (84.9)
Divorced/separated	8 (7.3)	1 (1.9)
Widowed/widowered	9 (8.3)	0
Living arrangement, *n* (%)		
Alone	10 (9.2)	5 (9.4)
With family	99 (90.8)	48 (90.6)
Type of stroke, *n* (%)		
Ischemia	75 (68.8)	
Haemorrhage	34 (31.2)	
Years since stroke (y), mean (SD)	6.58 (4.30)	
Hemiplegic side, *n* (%)		
Left	49 (45.0)	
Right	60 (55.0)	
FMA-LE, mean (SD)	24.45 (5.47)	
TUGT, mean (SD)	16.14 (12.51)	
CIM-C, mean (SD)	39.87 (7.56)	
PCS, mean (SD)	38.61 (10.19)	
MCS, mean (SD)	49.23 (10.83)	

n: number; BMI: body mass index; FMA-LE: Fugl-Meyer Assessment of Lower Extremity; TUGT, Timed Up-and-Go Test; CIM-C: the Chinese version of Community Integration Measure; PCS: physical component summary; MCS: mental component summary.

**Table 2:** Content validity index of the Chinese (Cantonese) version of the Brief 2-Way SSS.

Item	Expert A	Expert B	Expert C	Expert D	Expert E	Expert F	Item-level content validity index
1.	4	4	4	4	4	4	1
2.	4	4	4	4	4	4	1
3.	4	4	4	4	4	4	1
4.	4	4	4	4	4	4	1
5.	4	4	3	2	3	2	0.67
6.	4	4	4	4	4	4	1
7.	4	4	4	4	4	4	1
8.	3	3	3	3	3	3	1
9.	4	4	4	4	4	4	1
10.	4	4	4	4	4	4	1
11.	4	4	4	4	4	4	1
12.	3	3	3	3	3	3	1
Scale-level content validity index/mean							0.97
Total agreement							11
Scale-level content validity index/universal agreement							0.92

**Table 3:** Internal consistency of the Brief 2-Way SSS-C.

Item no.	Item	Corrected item-total correlation	Cronbach's alpha if item is deleted
Receiving emotion support: 0.88			
6	There is someone in my life I can get emotional support from	0.74	0.85
9	When I am feeling down, there is someone I can lean on	0.82	0.78
10	There is at least one person that I can share most things with	0.75	0.75
Giving emotion support: 0.85			
3	People confide in me when they have problems	0.83	0.68
5	I give others a sense of comfort in times of need	0.68	0.82
7	People close to me tell me their fears and worries	0.66	0.84
Receiving instrumental support: 0.87			
1	If stranded somewhere there is someone who would get me	0.74	0.84
11	I have someone to help me if I am physically unwell	0.76	0.82
12	There is someone who can help me fulfil my responsibilities when I am unable	0.78	0.80
Giving instrumental support: 0.74			
2	I help others when they are too busy to get everything done	0.55	0.66
4	I am a person others turn to for help with tasks	0.61	0.58
8	I have helped someone with their responsibilities when they were unable to fulfil them	0.52	0.69

**Table 4:** The results of test-retest reliability.

Item	Mean 1	Mean 2	ICC	95% CI low	95% CI high
1	2.67	2.57	0.77	0.64	0.85
2	2.52	2.45	0.76	0.64	0.85
3	2.69	2.51	0.79	0.68	0.87
4	2.25	2.24	0.72	0.59	0.82
5	2.69	2.72	0.63	0.46	0.75
6	2.96	3.00	0.66	0.50	0.78
7	2.84	2.79	0.75	0.62	0.84
8	2.46	2.51	0.60	0.42	0.74
9	2.84	2.70	0.69	0.54	0.79
10	3.03	2.93	0.66	0.50	0.77
11	3.16	3.18	0.59	0.40	0.72
12	2.93	2.84	0.73	0.59	0.82
Receiving emotional support	8.82	8.63	0.76	0.64	084
Giving emotional support	8.21	8.01	0.77	0.65	0.85
Receiving instrumental support	8.58	8.58	0.81	0.70	0.88
Giving instrumental support.	7.24	7.19	0.78	0.67	0.86

ICC: intraclass correlation coefficient; CI: confidence interval.

**Table 5:** Correlations between Brief 2-Way SSS-C and FMA-LE, TUGT, CIM-C, and SF12-C.

	Receive emotional support	Give emotional support	Receive instrumental support	Give instrumental support
FMA-LE	*r* = 0.21, *p* = 0.028^∗^	*r* = 0.36, *p* < 0.001^∗^	*r* = 0.23, *p* = 0.016^∗^	*r* = 0.36, *p* < 0.001^∗^
TUGT	*r* = −0.074, *p* = 0.441	*r* = −0.22, *p* = 0.024^∗^	*r* = −0.094, *p* = 0.33	*r* = −0.39, *p* < 0.001^∗∗^
CIM-C	*r* = 0.31, *p* = 0.001^∗∗^	*r* = 0.45, *p* < 0.001^∗∗^	*r* = 0.39, *p* < 0.001^∗^	*r* = 0.46, *p* < 0.001^∗∗^
PCS	Rho = −0.01, *p* = 0.91	Rho = 0.22, *p* = 0.023^∗^	Rho = 0.08, *p* = 0.413	Rho = 0.36, *p* < 0.001^∗∗^
MCS	*r* = 0.25, *p* = 0.008^∗^	*r* = 0.22, *p* = 0.023^∗^	*r* = 0.28, *p* = 0.004^∗^	*r* = 0.35, *p* < 0.001^∗∗^

^∗^ *p* < 0.05. ^∗∗^*p* < 0.001. FMA-LE: Fugl-Meyer Assessment of Lower Extremity; CIM-C: Chinese version of the Community Integration Measure; TUGT: Timed Up-and-Go Test; PCS: physical component summary; MCS: mental component summary.

**Table 6:** Comparison of Brief 2-Way SSS-C scores between stroke participants and healthy participants.

	Stroke participants (*n* = 109)	Healthy participants (*n* = 53)	*t* (*p* value)
Receiving emotional support, mean (SD)	8.91 (2.53)	10.87 (3.54)	-3.61 (*p* = 0.001)
Giving emotional support, mean (SD)	8.54 (3.10)	10.36 (2.67)	-3.85 (*p* < 0.001)
Receiving instrumental support, mean (SD)	8.89 (2.93)	10.09 (3.55)	-2.14 (*p* = 0.04)
Giving instrumental support, mean (SD)	7.57 (2.88)	10.17 (2.59)	-5.77 (*p* < 0.001)

**Table 7:** Mean Brief 2-Way SSS-C subscale scores of stroke participants with different characteristics.

Total sample (*n* = 109)	Receiving emotional support, mean (SD)	Giving emotional support, mean (SD)	Receiving instrumental support, mean (SD)	Giving instrumental support, mean (SD)
Sex, *t* (*p* value)	-0.52 (0.60)	-0.95 (0.34)	-1.56 (0.12)	-1.31 (0.19)
Women (*n* = 46)	9.65 (3.53)	9.17 (3.71)	9.89 (3.35)	8.54 (3.73)
Men (*n* = 63)	9.27 (4.12)	8.49 (3.65)	8.86 (3.51)	7.60 (3.67)
Education level, *F* (*p* value)	1.19 (0.31)	0.38 (0.68)	0.45 (0.64)	0.70 (0.50)
Primary school or below (*n* = 24)	10.42 (3.68)	8.21 (3.72)	9.75 (3.57)	7.63 (3.75)
Secondary school (*n* = 70)	9.27 (3.99)	8.97 (3.69)	9.27 (3.61)	8.30 (3.72)
College or above (*n* = 15)	8.60 (3.46)	8.80 (3.73)	8.67 (2.64)	7.20 (3.71)
Marital status, *F* (*p* value)	0.64 (0.59)	0.75 (0.52)	0.15 (0.93)	1.11 (0.35)
Single (*n* = 11)	9.00 (3.52)	7.91 (4.28)	9.00 (3.85)	6.91 (3.18)
Married (*n* = 81)	9.33 (4.00)	8.68 (3.67)	9.26 (3.53)	7.93 (3.73)
Divorced/separated (*n* = 8)	9.13 (4.29)	9.38 (4.34)	9.25 (3.69)	8.13 (4.85)
Widow/widower (*n* = 9)	11.11 (2.57)	10.22 (2.17)	10.00 (2.65)	9.89 (2.80)
Living arrangement, *t* (*p* value)	-0.59 (0.57)	-1.52 (0.16)	-0.41 (0.69)	-1.13 (0.29)
Alone	8.60 (4.77)	6.70 (4.64)	8.80 (4.10)	6.40 (4.81)
With family	9.52 (3.78)	8.99 (3.53)	9.34 (3.42)	8.16 (3.57)
Mobility function, *t* (*p* value)	-1.39 (0.17)	-3.27 (0.003)∗	-1.02 (0.31)	-3.08 (0.004)∗
Low level (FMA-LE<21) (*n* = 22)	8.41 (3.85)	6.45 (3.80)	8.64 (3.35)	6.14 (3.01)
High level (FMA-LE ≥21) (*n* = 87)	9.69 (3.85)	9.37 (3.42)	9.46 (3.50)	8.47 (3.74)

^∗^ *p* value < 0.05. FMA-LE: Fugl-Meyer Assessment of Lower Extremity.

## Data Availability

The data that support the findings of this study are available on request from the corresponding author.
